# Sports Action Recognition Based on Deep Learning and Clustering Extraction Algorithm

This article has been retracted.

**DOI:** 10.1155/2022/4887470

**Published:** 2022-03-19

**Authors:** Ming Fu, Qun Zhong, Jixue Dong

**Affiliations:** ^1^School of Science, Heilongjiang Bayi Agricultural University, Daqing, Heilongjiang 163316, China; ^2^School of Foreign Languages, Northeast Petroleum University, Daqing, Heilongjiang 163000, China

## Abstract

This paper constructs a sports action recognition model based on deep learning (DL) and clustering extraction algorithm. For the input detection image frame, athletes' movements are detected through DL network, and then athletes' sports movements are fused. Moreover, it expands new knowledge and improves learning ability through automatic learning training set. The neural network (NN) is applied to the sample set containing images of nonathletes, and the negative training sample set is iteratively enhanced according to the generated false positives, and the results are optimized by clustering method. Simulation experiments show that compared with other algorithms, the clustering extraction algorithm in this paper has achieved superior performance in recognition rate and false alarm rate, and the recognition speed is faster. The aim is to extract the athletes' training postures through the analysis of sports movements, so as to assist coaches to train athletes more professionally and provide some reference for sports movement recognition.

## 1. Introduction

At present, the level of science and technology of competitive sports training in China is relatively low, and the teaching method based on subjectivity and experience is generally adopted. With the naked eye and experience of coaches, athletes can only master the technical essentials through repeated exercises [1]. In intelligent monitoring, advanced human-computer interaction, automatic tagging, 3D games, medical diagnosis, and other aspects, the research of motion recognition has a wide application prospect and potential economic value [2]. Due to the diversity of sports movements, noisy scenes, changeable camera motion angle, and other characteristics, it is more difficult to recognize movements. Among them, the skeleton motion sequence is favored by the researchers of motion recognition because of its concise expression of motion mode and insensitivity to light and background [3]. However, the current research based on skeleton sequence mostly starts with extracting global motion features or uses local features to do motion recognition, which makes the detailed motion features easily overlooked [4]. There are some restrictive problems in traditional motion recognition, such as sensitive lighting, high cost, special equipment, and privacy intrusion. Therefore, the research of sports action recognition is still facing great challenges.

Motion recognition is widely used in many fields. Such as human-computer interaction, motion capture analysis, video monitoring and safety, environmental control monitoring, and prediction [5]. As an application direction of video data analysis, video-based motion recognition can automatically identify the motion in the video by computer after obtaining the video motion data, thus revealing the behavior of objects in the video [6]. The data source of motion recognition is not only video data but also depth images and bone motion data and even sensor data of smart devices can be used for motion recognition. With the rapid development of depth cameras and sensors, it is easier to acquire depth images and bone motion data, and motion recognition based on depth images and bone data has become a hot research field [7]. Detecting and tracking athletes in sports videos can obtain athletes' sports parameters, analyze athletes' behavior characteristics, and judge the standardization of athletes' actions, which is a necessary step for analyzing sports videos. Through the target detection and tracking of the game video, professionals can get the relevant data they need [8, 9]. The existing research needs too many features, and the recognition speed is slow, which cannot meet the real-time requirements well. Therefore, this paper proposes a sports action recognition method based on deep learning (DL) and clustering extraction algorithm.

Action recognition, as a basic part of behavior analysis, is a classification study of action category recognition at the action level. Human motion can be abstracted at different levels, so as to study human motion according to different levels [10, 11]. DNN has the ability of representation learning, and it has better performance than traditional computer vision technology and expert system in the fields of target detection and recognition, natural language processing, and so on. In view of the deficiency of existing research, this paper proposes a new method of sports action recognition. A test data set composed of athletes' images is established to verify the generalization ability of the network in the learning stage, and the optimal weight configuration is selected. The test set remains unchanged in the algorithm iteration. For neurons, clustering extraction algorithm is used to train the network and realize the detection of athletes' sports movements. The experimental results show that the sports action recognition method based on DL and clustering extraction algorithm proposed in this paper have good performance.

## 2. Related Work

Literature [12] extracted the shape and motion features, then matched them with the templates in the training set, and finally used the similarity vector as the input of SVM for recognition. Literature [13] uses a feedforward hierarchical network model to extract features and then uses SVM classification for action recognition. Literature [14] proposed an action recognition based on contextual information, using a bag-of-words model to represent scenes and actions, and finally using an SVM-based scene and action joint classifier for action recognition. Literature [14] proposed an algorithm for hiding conditional random fields, which was applied to gesture and head movement recognition. Literature [15] proposed a hierarchical CRF model and then combined with a hierarchical Gaussian latent variable model for 3D model human behavior recognition. Literature [16] proposed an action recognition model of attention mechanism based on time dimension. The time attention mechanism is added to the improved 3D convolution model. Literature [17] uses improved CNN to identify the fusion of bone information and depth information and designs a sports action recognition test system based on Kinect and MATLAB and establishes a virtual learning environment-oriented action database to verify the feasibility of the algorithm. Literature [18] proposed a new representation method of bone sequence. The bone sequence is converted into a data structure similar to the image so that the VGG network can be used to extract the temporal features of the motion, and then a multitask learning network is introduced to jointly process these features and absorb the spatial structure information. Literature [19] calculated five-dimensional feature vectors based on human body parts, and then clustered them based on the feature vectors, and extracted the motion features of related joint positions from the clustered clusters. K-means clustering method is used to obtain K poses. The action graph is constructed based on these postures, and the recognition result is obtained using maximum likelihood estimation based on the action graph. Literature [20] proposed an action recognition model based on bone-based graph convolutional network. It is the first time that graph convolution is applied to bone-based action recognition. The paper describes the convolution operation on the graph, considering the convolution operation in the first-order neighborhood and, at the same time, defines three adjacent point division labeling methods to encode the graph. It can show the change information of the vertices. Literature [21, 22] summarizes the current research status of human motion recognition, including video-based, sensor-based, and radio-frequency-based research status. Literature [23] analyzed the basic principles of CNN and established a structure based on CNN. Then, the action database is randomly allocated into training samples, verification samples, and test samples. Use training samples and verification samples to train and verify the model, and then use the test samples to test the model, and finally get the classification accuracy of different actions. Literature [24] proposed a moving target detection method based on U-NetDL network. Experimental results show that the algorithm only needs fewer frames of images as the training set to obtain extremely high detection accuracy, and the detection results will not be significantly biased toward moving objects or the background. Literature [25] proposed a DL-based human action recognition method. The key technology of human action recognition is analyzed. Based on previous research, this paper proposes a new method of sports action recognition. The features are extracted from the rectangular images of athletes, and then a strong classifier is constructed to extract the static features, dynamic features, and compensation features of the bone information as effective bone features, and use optimized deep belief network recognition; at the same time, change the number of joint points to verify the impact on action recognition, and further extract the depth features and skeletal features of the action, and use DNN for recognition to obtain the best recognition effect and robustness. Its model has achieved good performance in sports action recognition [26].

## 3. Methodology

### 3.1. Action Recognition Research

Human action is a nonverbal communication method. Human actions can be used instead of language to express specific meanings in specific situations. There are three types of commonly used motion data: color images, depth data, and bone data. The essence of human action recognition is to obtain classification results through learning video data or image sequences [27]. Sports action recognition research is generally an experimental test conducted on a public database to verify the feasibility of the method. Normally, the action data in the database is subjected to simple preprocessing after the action is extracted, such as denoising and background removal.

From preprocessing to feature selection, the sports action information is extracted from the underlying data, and then the category is marked by the classifier to complete the action recognition. The process of action recognition is to obtain high-level action information through the bottom data, so as to learn the action characteristics and finally realize the process of action classification [28]. Good feature expression is critical to the final accuracy of the algorithm. The calculation and testing of various pattern recognition algorithms are mainly reflected in the feature extraction stage, which takes the most time. Therefore, feature extraction is critical to the accuracy of sports action recognition. The division of motion representation is shown in Figure 1.

The movement characteristics are spatiotemporal; different from the texture and edge features extracted from image data, this two-dimensional feature pays attention to the spatial distribution of pixels, while the motion features have dual characteristics of time and space. Timeliness is manifested in that the motion features pay attention to the motion pattern of the moving subject with the passage of time, and the motion is very rich in shape and motion changes, and the quality of motion features directly affects the accuracy of recognition. Therefore, motion feature extraction is a crucial link in sports motion recognition [29]. The former mainly extracts the spatial features directly, while the latter mainly uses the position coordinates, angles, and other features of the skeleton joints that represent the outline of human body.

After selecting motion features, the next step is to generate a motion recognition model, that is, to design a classifier. Even if good features are extracted, there is no guarantee that the recognition result will be good. Only by designing a matching classifier and combining them perfectly can we get considerable recognition results. The feature recognition process is largely regarded as a supervised classification process, assuming that the number of action categories and the sample sets of known categories are determined. In the training stage, these sample sets are used to generate the sports action recognition model, and then the model can be used for the actual test in the recognition stage.

Classification refers to mapping data records into a given category by using classification functions or constructed classification models on the basis of existing data. Classifier is very important for data prediction and one of the important methods of data mining. Common motion recognition classifiers can be divided into two categories according to the extracted features: one based on time series features and the other based on fixed dimension features. By dividing the image into regions, the amount of information in the image can be effectively reduced, the amount of data to be processed in the subsequent steps of the algorithm can be reduced, and the computational burden can be significantly reduced. Compared with drawing fixed static grids on different images, using superpixel algorithm to divide regions on different images has obvious advantages, because compared with fixed static networks, superpixel algorithm can identify object boundaries more accurately so that the color intensity of each region can be as same as possible so that the subsequent feature extraction work can be carried out more smoothly.

### 3.2. DL and Clustering Extraction Algorithm

DL is a branch of machine learning, which has made great breakthroughs in application such as speech recognition, computer vision, and image classification in recent years. Its principle is to simulate the neurons of the human brain by establishing a model. When you see images or receive text and audio information, you can express the data through multilevel features and finally understand the data. When observing an image, the processing sequence of brain neurons on the image is as follows: edge information, initial shape, and finally complete image information. The principle of DL is to simulate the combination of human neurons from low-level features to high-level features, so as to describe and understand objects. The structure of single layer perceptron is shown in Figure 2.

Similar to the process of human brain recognizing objects, DL is to form more abstract high-level features by combining the features of the bottom layer. Take the face as an example. First, the low-level features of DL are edge features, that is, edges in a certain direction in the image. Then, we learn the combined pattern of these edge features and get local intermediate features, such as the eyes and nose. Finally, the basic patterns are combined to form advanced features corresponding to the whole face image.

The feature of neural network (NN) is that the original image can be directly used as the network input, unlike the traditional algorithm which needs to extract features manually, the method of local interconnection makes the obtained features independent of translation, scaling, and rotation, and the method of weight sharing also greatly reduces the number of parameters, thus reducing the complexity of the model and improving the training efficiency. In order to reduce the dimension of features, the downsampling method uses the characteristics of local association to sample the local areas of the feature map. NN is an operational model, a simple model based on the abstraction of human brain neuron network from the perspective of information processing and a network composed of multiple neurons connected in some form. The basic unit of NN is neuron.

### 3.3. Sports Action Recognition Model Based on DL and Clustering Algorithm

In reality, the pixels occupied by moving objects are far less than those occupied by the background, which will lead to common sample imbalance. This is a challenge to apply DL to the field of sports movement detection. Therefore, when processing training data, we should attach weights to samples to balance them. Most researchers express the posture of the human body by the outline or silhouette of the human body, express the boundary shape of the object by the contempt of the context, and identify it by applying the shape context.

In DL, before inputting data into NN for training, there is usually a process of data preprocessing and conversion. Given a set of samples {(*x*^(*i*)^, *y*^(*i*)^)*|*1 ≤ *i* ≤ *N*}, the output of NN is f(x w, b). NN is propagated in the following formulas:

(1) $$\begin{array}{c} z^{\left(l\right)}=W^{\left(l\right)}\cdot a^{\left(l-1\right)}+b^{\left(l\right)}, \end{array}$$

(2) $$\begin{array}{c} a^{\left(l\right)}=f_{l}\left(z^{\left(l\right)}\right). \end{array}$$

The objective function is

(3) $$\begin{array}{c} J\left(W,b\right)=\sum_{i=1}^{N}L\left(y^{\left(i\right)},f\left(x^{\left(i\right)}|W,b\right)\right)+\frac{1}{2}\lambda {\left\|W\right\|}_{F}^{2}\\ =\sum_{i=1}^{N}J\left(W,b;x^{\left(i\right)},y^{\left(i\right)}\right)+\frac{1}{2}\lambda {\left\|W\right\|}_{F}^{2},\\ {\left\|W\right\|}_{F}^{2}=\sum_{l=1}^{L}\sum_{j=1}^{n^{l+1}}\sum_{j=1}^{n^{l}}W_{ij}^{\left(l\right)}. \end{array}$$

Among them, *n*^(*l*)^ represents the number of neurons in the first layer; *f*_*l*_(·) represents the activation function of layer *l*; *W*^(*l*)^ represents the weight matrix from the l-1th layer to the lth layer; *b*^(*l*)^ represents the offset from the l-1th layer to the lth layer; *z*^(*l*)^ represents the state of neurons in the first layer; *a*^(*l*)^ represents the activity value of the first layer of neurons; W and *b* are the weight matrix and bias vector containing each layer. For the first layer, define an error term, as shown in the following formula:

(4) $$\begin{array}{c} \delta^{\left(l\right)}=\frac{\partial J\left(W,b;x,y\right)}{\partial z^{\left(l\right)}}\in R^{n^{\left(l\right)}}. \end{array}$$

Its mathematical meaning is the partial derivative of the objective function with respect to the neuron *z*^(*l*)^ of the first layer. The physical meaning is the influence of neurons in the first layer on the final error, that is, the sensitivity of the final output to the final error of neurons in the first layer.

Classification DNN is used, and fine-tuning is carried out on the sports posture image by using the model trained on the data set. When training the model, the initial parameters determine the training speed and the quality of the model. In the supervised training process of DL, if there is a serious imbalance in the number of samples in different classification categories, the category with fewer samples will have the phenomenon of “underlearning.” It may cause the trained model to tend to predict the unknown samples as a category with a large number of training samples. This is a common problem of classification bias. In the field of moving object detection, the classification categories are generally moving objects and background, and in reality, the pixels occupied by moving objects are far less than those occupied by background, which easily leads to the problem of classification bias.

For a multiclassification task with C classes, *r* score vectors are obtained after feature extraction with test samples, and their distances relative to the i-th class are calculated, respectively. It is recorded as *d*_*i*_^*j*^, *j* ∈ {1,2,…, *r*}, *i* ∈ {1,2,…, *C*}. The algorithm is as follows:

Calculate *β*_*j*_:

(5) $$\begin{array}{c} \beta_{j}=\frac{h_{j}-\min\left(d_{1}^{j},d_{2}^{j},\ldots ,d_{C}^{j},\right)}{h_{j}},\\ h_{j}=\sum_{i=1}^{C}d_{i}^{j}j\in \left\{1,2,\ldots ,r\right\}. \end{array}$$

Standardize *d*_*i*_^*j*^ to the interval [0,1]. For convenience, it is still recorded as *d*_*i*_^*j*^.

(6) $$\begin{array}{c} d_{\max}^{j}=\max\left\{d_{1}^{j},d_{2}^{j},\ldots ,d_{C}^{j}\right\},\\ d_{\min}^{j}=\min\left(d_{1}^{j},d_{2}^{j},\ldots ,d_{C}^{j},\right),\\ d_{i}^{j}=\frac{d_{\max}^{j}-d_{i}^{j}}{d_{\max}^{j}-d_{\min}^{j}}. \end{array}$$

Arrange *d*_*i*_^*j*^ in ascending order, and the result after arrangement is *e*_1_^*j*^ ≤ *e*_2_^*j*^ ≤ …≤*e*_*C*_^*j*^. Calculate *w*_*j*_.

(7) $$\begin{array}{c} w=\sum_{j=1}^{r}e_{2}^{j}-e_{1}^{j},\\ w_{j}=\frac{e_{2}^{j}-e_{1}^{j}}{w}. \end{array}$$

Since *e*_1_^*j*^=0, the above formula is simplified to

(8) $$\begin{array}{c} w=\sum_{j=1}^{r}e_{2}^{j},\\ w_{j}=\frac{e_{2}^{j}}{w}. \end{array}$$

Calculate *f*_*i*_:

(9) $$\begin{array}{c} f_{i}=\sum_{j=1}^{r}\beta_{j}w_{j}d_{i}^{j}. \end{array}$$

Let $k=\underset{i}{\arg}\max f_{i}$, and *k* is the classification label after the score fusion. From the above calculation process, it can be seen that the entire fusion method does not specify the setting of the weight parameter, and the *β*_*j*_*w*_*j*_ as the weight is calculated by the score vector. In this way, the weights can be flexibly set for the differences between different samples or different score vectors.

In DL, the increase of network depth makes the extracted features richer and the learning ability of the model stronger. On the other hand, the increase of depth makes the training of the model more difficult, and problems such as gradient explosion or gradient disappearance hinder the convergence of the model, which can be solved by standardization or regularization.

Generally, there are two ways to obtain fixed dimension features: one is to sample the original video sequence to obtain a fixed number of frames, which has a higher feature dimension; the other is to use histogram expression to extract low-level features from the whole video and cluster them to get a dictionary and then assign the features to the corresponding dictionary primitive histogram to represent the video features. Nowadays, the problem of motion recognition is mostly used for the feature representation of fixed dimensions, and most pattern recognition classifiers can be used for sports motion recognition. Divide and fine-tune the area. Traverse the image with the four corners of the image as the starting points in turn, and update the label value of each pixel point to the minimum value that is not 0 among the label values of four neighboring points until the label values of all points do not change any more.

The best way to solve the over-fitting problem is to choose the appropriate model capacity, so as not to make the model capacity too large to cause the over-fitting problem. The size of the model capacity depends on the use of the function selection space of the training algorithm in the model. DNN network extracts the features of the region of interest. Each video frame image of the whole video will output a classification probability and take the category with the largest classification result as the candidate key pose. Finally, the action key frames are finally determined by the key frame extraction strategy.

## 4. Result Analysis and Discussion

Human skeleton joint points represent the position coordinates of sports movements in three-dimensional skeleton coordinates, which not only show the shape of human parts but also describe the topological information of human bodies. Individual bone information has no specific meaning, but the relationship between them can be used as an effective feature of sports movements, and the recognition result will not be seriously affected by the change of distance from the camera and human objects, which has good robustness.

Besides the space size of convolution kernel, the size of time dimension also affects the classification and recognition rate. According to the research, when the time dimension is 3, the final classification and recognition accuracy is higher. For the choice of pool core size, according to the purpose of pool, the dimension and resolution of feature surface are reduced to avoid premature over-fitting. The size of the pool core of each pool layer should be set based on the convolution result size of its convolution layer. If the pool core is too large, some action information will be lost, and if the pool core is too small, it canno't achieve the due pool purpose.  Figure 3 is a comparison of segmentation accuracy of sports motion recognition with convolution kernels of different sizes.

By analyzing the movements in the database, it is found that these movements have a large amplitude and are not as detailed as the joints such as wrists and ankles, so eliminating these joints has little effect on the recognition rate. However, when the movements are delicate, involving joints such as wrists and ankles, which are not easy to distinguish, these joints are very important for the recognition of movements and cannot be eliminated. Although eliminating these joint points will improve the calculation efficiency, when these joint points have a great influence on the recognition results, the method of improving the calculation efficiency at the expense of the recognition rate is not in line with the original intention of the experiment, and this method is not desirable. Experiments were conducted on two datasets, and the experimental results were presented and evaluated. The changes of the training error and test error of the model on two datasets are shown in Figures 4 and 5.

It can be seen from the figure that after the model reaches convergence, it can reduce the training error and test error to varying degrees. Before adding residual error, there is a certain gap between the test error and the training error of the model, which is because the generalization ability of the model among individuals is weak, while after adding residual structure, the gap between the training error and the test error is narrowed, which shows that the residual structure strengthens the generalization ability of the model among subjects and the performance of the model is further improved.

In order to improve the recognition accuracy and effect, the depth features and bone features of depth information and bone information are extracted, respectively, and feature fusion is carried out. After feature fusion, the improved NN is used for recognition to obtain the best recognition effect and robustness. In this paper, because we deal with the nongridded bone motion data, there are not many bone joint points on the spatial scale, and the spatial scale is smaller after dividing the bone joints, and the convolution added to the spatial dimension does not need a full connection layer to combine the joint spatial features. Therefore, after the global spatiotemporal pooling, this paper introduces two full connection layers to map the hidden layer motion features to the score vector space, which acts as a classifier.

In the experiment, the correlation of three-dimensional coordinates between bone nodes is extracted as the bone features of sports, and the features are identified by DNN for classification. Finally, the algorithm is applied to three motion subsets of MSRAction3D database for experiments, and the influence of the number of bone joint points on the motion recognition rate is compared. The recognition result is shown in Figure 6.

As can be seen from Figure 6, test 2 has the best recognition effect. The reason is that the proportion of training set data in test 2 is more than that in test set data, and one of the characteristics of DL is its strong learning ability. During the training process, the model learned more experience. It can be seen that the more the training data, the better the learning situation and the better the recognition results.

In order to effectively evaluate the model in this paper, many aspects are fully considered, and the model is compared and tested. The recognition accuracy between this model and traditional model and gated recursive convolution network is shown in Figure 7. The comparison of recognition speed is shown in Figure 8.

In the model, the spatial features and temporal features of sports action recognition are simultaneously learned, that is, the features of each frame of video are learned by 2DNN, and then the time series between frames is learned by the corresponding cyclic NN unit, and finally the results are obtained by softmax classifier. It can be seen from the figure that compared with the other two models, this model improves the recognition accuracy of sports movements, reduces the running time, and improves the recognition speed to a certain extent.

The experimental results show that this method only needs a small amount of training data to obtain an excellent network model. Moreover, the trained model can achieve extremely high detection accuracy. After using weight to adjust uneven samples, the detection results are not obviously biased towards moving objects or background. Compared with traditional methods, the detection results of this method are more accurate and the recognition speed is faster.

## 5. Conclusions

In the past research, most researchers focused on the global motion feature acquisition and identified the motion samples based on the global motion features. This paper introduces the related knowledge of DL. DL is a deep model, which has strong analysis and processing ability for complex problems and good generalization. This paper puts forward a sports action recognition method based on DL and clustering extraction algorithm, which starts with the motion characteristics of local parts to recognize the action samples. From the aspect of feature extraction, sports action recognition algorithms are divided into two categories: non-DL-based methods and DL-based methods, and they are introduced in detail. The non-DL method relies too much on artificial prior knowledge, which requires higher sports action video library. The method of DL has good adaptability to sports action video library and can learn action information better and get better representation. The proposed method is compared with the methods in other papers to verify the feasibility of the proposed algorithm. Experiments show that the algorithm has good recognition and robustness. The recognition efficiency is high and the time is short.

## Figures and Tables

**Figure 1:** Motion representation partition.

**Figure 2:** Single layer perceptron network structure.

**Figure 3:** Comparison of segmentation accuracy of sports action recognition based on convolution kernels of different sizes.

**Figure 4:** Error variation of the model on UTD-MHAD data set.

**Figure 5:** Error variation of the model on NTU-RGB + *D* data set.

**Figure 6:** Recognition rate of bone information.

**Figure 7:** Comparison of model recognition accuracy.

**Figure 8:** Model identification speed comparison.

## Data Availability

The datasets used and/or analyzed during the current study are available from the corresponding author on reasonable request.
